# Transient Cardiac Dysfunction in Cerebrovascular Accidents

**DOI:** 10.7759/cureus.10185

**Published:** 2020-09-01

**Authors:** Ahmed Elkhouly, Rana A Tauseen, Steven Hamilton, Sara L Wallach, Adam C Kaplan

**Affiliations:** 1 Internal Medicine, St. Francis Medical Center, Trenton, USA; 2 Medicine, St. Francis Medical Center, Trenton, USA; 3 Internal Medicine, Hackensack Meridian School of Medicine at Seton Hall University, Nutley, USA

**Keywords:** cerebral t waves, left ventricular systolic dysfunction, acute cerebrovascular accidents

## Abstract

Acute cerebral injuries have been repeatedly correlated with sudden and different electrocardiogram (EKG) changes, such as cardiac arrhythmias, QT prolongation, and abnormal T-wave morphology. One rare phenomenon is “cerebral T-waves,” which are T-waves observed in the context of stroke and described as transient, symmetric, and deeply inverted. Moreover, few studies linked acute cerebral injuries with transient cardiac dysfunction secondary to autonomic dysfunction.

The classic cerebral T-waves are defined as a T-wave inversion of ≥5 mm depth in ≥4 contiguous precordial leads, and it is more commonly observed in the setting of acute ischemic stroke rather than hemorrhagic stroke. We present a patient who presented with acute pulmonary edema, T-wave inversions in the precordial leads, and left ventricular (LV) dysfunction initially suspicious for acute coronary syndrome (ACS). However, computer tomography of the brain performed on the third day of his hospital stay proved us wrong.

## Introduction

T-wave changes on electrocardiogram (EKG) may be the result of various conditions that might be cardiac or non-cardiac in origin. The differential diagnosis for these changes is overwhelmingly cardiovascular in origin but neurologic etiologies are well documented. Cardiovascular etiologies of T-wave changes include myocardial ischemia, myocardial infarction, myocarditis, pericarditis, and ventricular hypertrophy with strain pattern. Neurologic causes include subarachnoid hemorrhage, subdural hematoma, and acute cerebrovascular accidents (CVAs) [1]. Cerebral ischemic or hemorrhagic events have been associated with various EKG changes with the most frequent being transient, deep, symmetric inverted T-waves in the precordial leads. The exact mechanism for the development of these “cerebral T-waves” is not well established but a few studies hypothesize possible injuries to the insular cortex. This injury would result in an increase in sympathetic tone to the cardiac system resulting in the observed changes [2]. One recent retrospective study even went beyond the transient EKG changes and linked acute cerebral injuries with a transient reduction in systolic function, due to autonomic dysfunction, which further expands on the potential role of central nervous system insult resulting in cardiac anomalies [3].

## Case presentation

We present a 75-year-old male patient with a past medical history of diabetes mellitus and an unremarkable family history who presented to our emergency department (ED) after the sudden onset of shortness of breath and sweating witnessed by his friend. During transport to the hospital, the patient's shortness of breath worsened with accompanying hypoxia. Conservative measures to support his respirations failed and he was intubated in the field. In the ED, the patient was found to be hypertensive with a blood pressure of 173/92 mmHg, heart rate of 82 beats/min, diffuse inspiratory fine crackles on auscultation with markedly elevated venous jugular distention. The rest of his physical examination was unremarkable, albeit limited secondary to the patient being sedated and intubated. Discussion with his friend did not reveal a history significant for chest pain at the time of symptom onset. Blood work was remarkable for highly elevated B-type natriuretic peptide (BNP) of 2943 pg/mL (< 100 pg/mL) and troponin I of 0.09 ng/mL (<0.03 ng/mL), hemoglobin A1c of 7.1 %, total cholesterol of 153 mg/dL, low-density lipoprotein (LDL) of 111 mg/dL, and negative urine drug screen. The remainder of his blood work was unremarkable. In the ED, the chest X-ray was remarkable for increased bronchovascular markings suggestive of pulmonary edema, EKG showed T-wave inversions in the pericordial leads from V1 to V5 (Figure 1), and CT scan of the brain without contrast was unremarkable for any ischemic or hemorrhagic pathology.

**Figure 1:** EKG showing T-wave inversions over the precordial leads (black arrows).

Due to his initial presentation with acute pulmonary edema, elevated troponin levels, and T-wave inversions in the EKG, the patient was treated for acute coronary syndrome with aspirin, high-intensity statin, intravenous heparin drip, and intravenous diuretics. Troponin follow-up showed a peak of 1.88 ng/mL. Emergent echocardiography showed moderately reduced left ventricular systolic function, an ejection fraction of 40-45%, with hypokinesis-akinesis of the mid and basal inferior wall segment with no evidence of left ventricular wall thrombus. Due to the critical nature of the patient cardiology deferred coronary angiography until the patient was more stable. However, on day 3 of the hospital course, a detailed neurological examination revealed areflexia, an up-going Babinski sign, and decreased motor strength affecting the proximal and distal muscle groups of his right upper and lower extremities.

Secondary to this finding, a CT-head was ordered which revealed a large evolving infarct within the left temporal/parietal lobe (Figure 2). Interestingly, repeat EKG’s showed resolution of the previously identified T-wave inversions (Figure 3). Upon multidisciplinary discussion, it was determined that his clinical presentation, particularly the reversible T-waves in four contiguous leads and wall motion abnormalities, was likely due to his large ischemic infarct and not likely due to the acute coronary syndrome, and therefore, the patient did not undergo coronary angiography during his hospitalization and was deferred by cardiology for outpatient workup. Unfortunately, the patient was lost to follow-up.

**Figure 2:** CT scan on the third day of admission showing large evolving infarct within left temporal/left parietal lobe (yellow arrow).

**Figure 3:** EKG showing the resolution of the T-wave inversions on the third day of hospital stay (black arrow).

## Discussion

Cerebral T-waves and LV dysfunction are rare findings in patients with acute cerebrovascular events. A retrospective study done by Jeremy et al. showed that in 800 patients with an acute CVA, only 17 patients were found to have cerebral T-waves on EKG with the majority of cases involving the middle cerebral artery (MCA; 11 patients out of the 17). Furthermore, they went on to describe three patients with concurrent LV wall motion abnormalities and cerebral T-waves, who all had infarcts in the MCA distribution, similar to our patient’s findings [3]. Rogers et al. described the proposed pathophysiology behind an acute cerebrovascular event and cardiac dysfunction, and in their study, they stimulated the left stellate ganglion, where marked negativity of the T-waves was observed [4]. The findings of Rogers et al. paired with the role the insular cortex plays in autonomic regulation, which when disrupted from an MCA infarct, can lead to the cardiac abnormalities that provide an explanation for the observed presentation of our patient.

While, there is no debate that a patient presenting with pulmonary edema, EKG changes, and elevated troponins should be evaluated for ACS, we believe it is important to recognize other potential etiologies so delays in a correct diagnosis and unintentional treatment harm can be minimized. Examples of such harms may be the rapid lowering of blood pressure or initiating anticoagulation as indicated in ACS, but not for an acute ischemic stroke

We recognize our limitation in fully attributing the patient's presentation and EKG findings to his central nervous system event, as a cardiac catheterization was never performed. However, the importance of not anchoring to a diagnosis on initial presentation is a skill that all healthcare practitioners should be cognizant. The lack of chest pain, only a moderate rise in troponin, and resolution of the T-wave changes hinted at the possibility of other etiologies for our patient who only became clear upon follow-up examination when a focal neurologic deficit became apparent.

## Conclusions

Cerebral T-waves and LV dysfunction are rare presenting signs in cerebrovascular injuries, but the recognition of this entity is extremely important not only to mitigate potential unnecessary treatment harms to the patient but also to recognize the potential true etiology, stroke, and initiate early goal-directed stroke care.
